RETRACTED

# Feasibility and Application of Cluster Nursing to the Care of Patients with Acute Oncology

**DOI:** 10.1155/2022/8973449

**Published:** 2022-07-31

**Authors:** Jun Song, Lei Fu

**Affiliations:** Emergency Department 2, Shengjing Hospital Affiliated to China Medical University, Shenyang 110000, Liaoning, China

## Abstract

**Objective:**

To probe the utility of cluster nursing for the care of acute oncology clients.

**Methods:**

One hundred fourteen cases of acute oncology pioneers undergoing therapy in our clinic from April 2019 to February 2021 were randomly assigned into two consecutive arms, conventional care and cluster care, in accordance with the nursing modality. Complications, satisfaction, quality of survival, and negative emotions were compared across the two parties.

**Results:**

The comorbidity incidence rate of the subject matter in the research cohort was 7.02%, which was below the comorbidity rate of 17.54% in the reaction cohort (*P* < 0.05); the percentage of satisfaction in the research cohort was 96.49%, which was higher than the satisfaction rate of 78.95% in the reaction cohort (*P* < 0.05); aftercare, the quality of survival was significantly higher in both groups, and the SAS and SDS scores were significantly lower, with a more pronounced trend of change in the research cohort than in the reaction cohort (*P* < 0.05).

**Conclusion:**

Bundled care for casualty oncology is of major value, with a marked reduction in the incidence of postoperative complications, high quality of survival, an excellent prognosis and negative mood, high patient morale and satisfaction and compliance with curative treatment, and good support for subsequent care.

## 1. Introduction

Due to the particularity of the disease, long-term fear and stress in tumor patients will lead to depression and anxiety in the patients. In addition, due to the impact of tumor consumption on metabolism, patients will be accompanied by mental and consciousness disorders, and such people are more susceptible to susceptibility. Oncology surgery patients are usually treated with chemotherapy, in the process of chemotherapy through peripheral venous puncture central venous catheter (PICC) is more widely used, the pain caused by repeated puncture can be avoided, and at the same time can largely reduce the damage and stimulation of blood vessels [1]. Failure to do so can lead to a range of complications that can impact patient care and health status recovery [2]. To avoid complications during the indwelling of the PICC catheter and ensure the smooth progress of the treatment process, this study adopts the cluster nursing method, which has high application value in improving the prognosis of patients. It is an evidence-based nursing method. Effective collection can realize nurse-led and multidisciplinary team cooperation. The main concept of nursing is “all-around nursing,” which is helpful to relieve patients' negative emotions and improve the safety of treatment [3]. The application of this nursing approach has prolonged the time of PICC catheter placement and improved the quality of survival. This nursing approach has matured in foreign studies, and although it started later in China, it has now been reported in emergency and malignant tumors [4].

RETRACTED

In the current census, 114 emergency oncology patients treated in our institute from April 2019 to February 2021 were selectively selected to inspect the value of the application of clustering nursing, which is reported as follows.

## 2. Materials and Methods

### 2.1. General Materials

One hundred fourteen urgent oncology patients undergoing therapy in our clinic from April 2019 to February 2021 were selectively recruited. In the reference arm (*n* = 57), there were 32 males and 25 females, mean age was 46.32 ± 4.07 years, mean disease duration was 2.65 ± 0.34 years, mean BMI was 22.35 ± 2.04 kg/m^2^, and placement site: 3 left arms and 54 right arms; in the study group (*n* = 57), there were 33 males and 24 females, mean age was 46.33 ± 4.09 years, target age was 46.33 ± 4.09 years, mean disease duration was 2.64 ± 0.35 years, mean BMI was 22.32 ± 2.06 kg/m^2^, and site of cannulation: 2 cases in the left arm and 55 cases in the right arm. The data were comparable (*P* > 0.05), the patients were aware of the exercise, and the study was approved by the institutional ethics committee.

#### 2.1.1. Inclusion Criteria

(1) Pathologically diagnosed acute oncology patients; (2) patients requiring infusion or catheterization; (3) patients with no communication or functional impairment and consciousness; (4) adult recipients.

#### 2.1.2. Exclusion Criteria

(1) Organ failure; (2) end-stage disease; (3) hypercoagulable blood or thrombosis history; (4) coinfectious disorders.

### 2.2. Methods

#### 2.2.1. Routine Care

Nursing staff provided personal self-care guidance and health education to patients and dealt with adverse reactions such as allergies, infections, and blocked tubes in a timely manner during the care process.

#### 2.2.2. Clustered Nursing

(1) Skills and knowledge training: the cluster nursing team is established, and the members of the team are trained in practical and theoretical knowledge. Only after passing the assessment (theoretical and practical assessment scores are higher than 80 points) can they take on nursing work. (2) Health education: the movement of the arm and trunk on the side where the tube is placed should not be too great, patients should wear loose clothing when lying in bed as far as possible and avoid pressure on the limb on the side where the tube is placed when asleep, patients should perform fist-clenching and fist-unclenching movements from time to time, and if the patch does not fit the skin, the nursing staff should be informed promptly for replacement. The nursing process should also observe the patient's mood fluctuation condition, take the initiative to ask about the situation and subjective feelings of the patient in a gentle tone, and give support and encouragement to the patient. (3) Aseptic operation: nursing staff should pay attention to hand hygiene, nursing and puncture utensils should be disinfected before use, an iodophor, cotton balls, and swabs should be disposable and used as they are opened. (4) Standardize the catheterization process: assess the patient with the aid of ultrasound and select the appropriate catheterization vessel according to the patient's specific condition; the diameter of the cathetezised vessel needs to meet the requirement of greater than two times the diameter of the catheter, and deliver the tube at the appropriate speed, with any resistance being dilated with sodium chloride injection to reduce the resistance, but it is worth noting that mandatory tube delivery or repeated pumping is strictly forbidden. (5) Develop standards for maintenance of the catheter: daily replacement of the positive pressure connector, routine disinfection of the catheter connection, and also observation of the catheter patency and flushing by choosing the pulsatile positive pressure flushing method. The catheter scale is observed in detail and recorded during care so that catheter displacement can be judged. The catheter patch should be changed at least once a week, and after this is done, the patch should be removed from top to bottom and the puncture site disinfected, then the tension-free patch should be placed on the punctured skin and fixed effectively to ensure it is airtight, and the maintenance date and person should be written on the patch. The date of maintenance and the person who maintains it are written on the film. (6) Posthospital follow-ups: nursing staff gave discharged patients an instruction manual and conducted regular 3-month telephone follow-up to understand the maintenance status of catheters outside the hospital, continue to promote nursing work, improve patients' professional identity with nursing staff, and improve nursing satisfaction and compliance.

RETRACTED

### 2.3. Observation Indicators

#### 2.3.1. Complications

All subjects received prognostic follow-up, and no patients were lost to follow-up. Patients were monitored for a 3-month prognosis after care, and catheter obstruction, venous thrombosis, phlebitis, and other conditions were recorded. Phlebitis was graded into 4 levels according to the severity of the patient, with no obvious symptoms as level 0, redness or pain at the puncture site as level 1, redness and pain at the puncture site as level 2, redness and palpable striated veins at the puncture site with obvious pain as level 3, and redness and palpable striated veins at the puncture site with obvious pain and overflowing pus as level 3. There was a positive correlation between the incidence of adverse reactions and patient prognosis.

#### 2.3.2. Satisfaction

The hospital customized satisfactory scale was applied to assess patient satisfaction, with greater than 85 being very pleased, 65–85 being pleased, and less than 65 being dissatisfied [5]. Satisfaction = number of cases (very satisfied + satisfied)/total number of cases, multiplied by 100%.

#### 2.3.3. Quality of Survival

The quality of life was assessed using the interview method, which contains 6 functions: environment, physical functioning, social relationships, psychological status, independence, and religion/spirituality, with a total score of 100 [6]. The score is positively correlated with the quality of survival.

#### 2.3.4. SAS and SDS Scores

53 is the upper limit of the normal score, >70 is severe anxiety and depression, 63–72 is moderate anxiety and depression, and 53–62 is mild anxiety and depression [7]. SAS and SDS scores were positively correlated with patients' unhealthy moods.

### 2.4. Statistical Methods

It collects the data into EXCEL spreadsheet, SPSS22.0 statistics software is used for data analysis to collect data to carry out the normal distribution test, such as data conform to a normal distribution, count data are described by composition ratio and rate of complications, degree of satisfaction analysis of differences between groups, chi-square test, measurement data to (mean ± standard deviation), *T*-test was used to analyze the difference between the quality of life and negative emotion groups and *P* < 0.05 indicates that the difference between groups is statistically significant. GraphPadPrism8 was used in the study.

*(1) General Information of the Two Sets of Groups*. The gender, age, disease duration, and BMI of the two cohorts were not statistically significant (*P* > 0.05), indicating that the two groups of data are comparable, and the research feasibility is high (see Table 1) (Table 1). *(2) Simplification Ratio of the Two Complication Arms*. The occurrence of complex complications in the studied cohort was 7.02%, which was lower than that of the complication in the controversial category of 17.54% (*P* < 0.05) (Table 2 and Figure 1). *(3) Comparison of Satisfactory Level of Satisfaction between the Two Sets of Groups*. The degree of dissatisfaction in the case of the target date was 96.49%, which was above the control group's satisfaction rate of 78.95% (*P* < 0.05) (Table 3 and Figure 2). *(4) Survival Quality Contrast between the Two Teams.* Aftercare, the overall quality of survival was markedly higher in both arms, and the trend was more pronounced in the target arms than in the base arms (*P* < 0.05) (Table 4 and Figure 3). *(5) Comparison of SAS and SDS Scores between the Two Sets of Groups*. Aftercare, SAS and SDS scores were significantly lower in both groups, and the trend of lowering SAS and SDS scores was more evident in the control cohort (*P* < 0.05) (Table 5 and Figure 4).

RETRACTED

## 3. Discussion

The PICC method of intravenous drug delivery is often used clinically, which can reduce the degree of vascular irritation, the incidence of venous pressure is significantly reduced, the chance of drug extravasation is reduced, and there is little or no significant skin irritation or damage to the veins [8–10]. The PICC approach to intravenous drug delivery is becoming more widely used in malignancy treatment and has obvious advantages, but effective patient care is still required in the hope of ensuring chemotherapy continuity and reducing the impact on patient life safety [11–13]. Clustered care can standardize the steps of nursing operations and is a comprehensive nursing approach that can establish a good nurse-patient relationship and ideal patient care outcomes [14]. According to Tang [15], in the care of PICC tumor patients with tubes, adverse effects such as those caused by cluster care were substantially reduced, and the results of the two studies were highly similar.

Clustered care is a way of providing multiple elements of care in the same setting and, at the same time, is highly operational [16–18]. It is not just at the time of PICC placement, but throughout the entire care process after placement, so it needs to be applied with good rules of care, with clear goals and time characteristics [19]. All nursing staff need to have good nursing skills and undergo professional technical training before care, which guarantees the level and quality of care and enhances nursing safety and team care [20–22]. The results of this study showed that the satisfaction rate of the research group was 96.49%, which was 78.95% higher than that of the control group. Foreign scholars Liu et al. [23] researched the effect of cluster nursing in emergency tumors. The results showed that, after nursing, the patient satisfaction score was 95.37%. The results of this study are highly consistent with the results of foreign research. Therefore, this nursing method has high feasibility and has been well received by patients. The main guiding basis of cluster nursing is evidence-based medicine. Nursing staff can achieve good nursing through communication with patients, providing patients with more valuable nursing methods and achieving targeted nursing. For the improvement of patient outcomes, after nursing, the quality of life of patients was significantly improved, and the risk of infection was significantly reduced [24].

RETRACTED

The results of this study showed that the satisfaction rate of the study group was 96.49%, which was higher than the satisfaction rate of the check group, which was 78.95%, so it was said that the nursing care method was all highly feasible and achieved the unanimous praise of the patients [23]. The main guiding basis of intensive care is evidence-based medicine, and nursing staff can achieve good care by communicating with patients, can provide patients with more valuable care, can achieve targeted care, and can improve patient outcomes by integrating various elements, and after care, the quality of patient survival is significantly improved and the risk of patient infection is significantly reduced [24]. Oncology via patients with high psychological stress and loss of confidence in life and the application of the PICC catheter approach to intravenous infusion, where foreign bodies are implanted in the patient's body, can lead to physical discomfort symptoms, which disturbs the patient's life and aggravates anxiety [25]. By providing health education and psychological intervention to the patients, the nursing staff helped to relieve the patients' anxiety and depression and speed up the time of disappearing symptoms.

Cluster nursing is of great significance to the rehabilitation of emergency tumor patients, which can improve the negative emotions and prognosis of patients, and the satisfaction of patients and their families is high. The research can verify the feasibility and safety of the nursing method from three aspects of nursing staff, family members, and patients and can establish a friendly nursing model. Therefore, it is of practical significance to apply cluster nursing in the rehabilitation of emergency tumor patients in this study. However, the research will be affected by some confounding factors, so it cannot represent all the research results, and the research is only conducted on some groups, so the research results may be biased to a certain extent. In addition, the research is a single-center study, so it cannot be representative of the overall population. The promotion of this nursing method has had a certain impact. Therefore, it is necessary to conduct a multicenter and large-sample study based on the cluster nursing model, to extend the study period and to analyze the long-term prognosis effect of this nursing method on patients.

RETRACTED

## 4. Conclusion

Clustered care for emergency oncology patients is of great significance. The incidence of postoperative complications in patients is significantly reduced, the quality of survival is high, the prognosis and poor mood of patients can be effectively improved, and patient satisfaction and treatment compliance are high, which can provide good support for the next nursing work.

## Figures and Tables

**Figure 1:** Concurrent illnesses in both sets of groups. *Note*. In the evaluation of complications such as catheter detachment, catheter obstruction, venous thrombosis, local inflammatory reaction of the skin, and phlebitis, the incidence of complications in the study group was lower than that in the control group, and the difference between the groups was statistically significant (*P* < 0.05).

**Figure 2:** Satisfaction in both arms. *Note*. The research group was more satisfied than the control group, and the difference was statistically significant (*P* < 0.05).

**Figure 3:** Quality of survival in the two sets of groups. *Note*. In the evaluation of survival functions such as environment, physiological function, social relationship, psychological state, independence, and religion/spirit, the study group had a higher quality of life score than the control group, and the difference was statistically significant (*P* < 0.05).

**Figure 4:** SAS and SDS scores for both sets of groups. *Note*. There was no significant difference in SAS and SDS scores between the two groups before nursing, the negative emotions in both groups were significantly improved after nursing, and the difference was statistically significant (*P* < 0.05).

**Table 1:** General profile of the two cohorts.

Group	Number of examples	Gender (m/f)	Age (years)	Duration of illness (years)	BMI (kg/m^2^)
Control group	57	32/25	46.32 ± 4.07	2.65 ± 0.34	22.35 ± 2.04
Study group	57	33/24	46.33 ± 4.09	2.64 ± 0.35	22.32 ± 2.06
*X* ^2^/*t*	—	0.036	0.013	0.155	0.078
*P*	—	0.850	0.990	0.877	0.938

**Table 2:** Summary of complications in the two arms versus each other (cases, %).

Group	Number of examples	Catheter dislodged	Catheter blockage	Venous thrombosis	Local inflammatory skin reaction	Phlebitis	Incidence of complications
Control group	57	3 (5.26)	2 (3.51)	1 (1.75)	3 (5.26)	1 (1.75)	10 (17.54)
Study group	57	1 (1.75)	1 (1.75)	0 (0.00)	1 (1.75)	1 (1.75)	4 (7.02)
*X* ^2^	—	—	—	—	—	—	2.931
*P*	—	—	—	—	—	—	0.087

RETRACTED

**Table 3:** Contrast of contentment ratio between the two subgroups (cases, %).

Group	Number of examples	Very pleased	Satisfaction	Unsatisfactory	Satisfaction
Control group	57	31 (54.39)	14 (24.56)	12 (21.05)	45 (78.95)
Study group	57	43 (75.44)	12 (21.05)	2 (3.51)	55 (96.49)
*X* ^2^	—	—	—	—	8.143
*P*	—	—	—	—	0.004

**Table 4:** Quality of existence contrasted between the two arms ($\bar{x}\pm s$).

Group	Control group (minute)		Research group (minute)	
	Before nursing	After care	Before nursing	After care
Environment	12.14 ± 4.32	14.65 ± 5.42^a^	12.13 ± 4.35	18.48 ± 5.61^ab^
Physiological function	21.54 ± 6.71	24.62 ± 6.51^a^	21.52 ± 6.72	32.73 ± 8.61^ab^
Social relations	13.05 ± 4.17	16.22 ± 5.41^a^	13.29 ± 2.67	23.12 ± 6.35^ab^
Mental state	21.54 ± 6.52	25.43 ± 6.55^a^	21.73 ± 6.25	33.51 ± 8.24^ab^
Independence	15.52 ± 6.24	20.73 ± 6.67^a^	15.53 ± 6.21	30.91 ± 6.15^ab^
Religious/spiritual	20.12 ± 4.34	24.51 ± 4.72^a^	20.15 ± 4.33	28.63 ± 4.52^ab^

*Note.* ^a^ *P* < 0.05 means that there is statistical significance in the comparison within the group, and ^ab^*P* < 0.05 means that the difference is statistically significant in the comparison between the groups.

**Table 5:** Comparison of SAS and SDS scoring between the two sets of participants ($\bar{x}\pm s$).

Group	Number of examples	SAS score (minute)		SDS score (minute)	
		Number of examples	After care	Number of examples	After care
Control group	57	40.35 ± 6.85	32.57 ± 5.14^a^	40.68 ± 6.47	31.19 ± 5.23^ab^
Study group	57	40.36 ± 6.91	22.84 ± 4.21^a^	40.71 ± 6.42	21.76 ± 4.05^ab^
*t*	—	0.008	11.057	0.025	10.776
*P*	—	0.994	＜0.001	0.980	＜0.001

*Note.* ^a^ *P* < 0.05 means that there is statistical significance in the comparison within the group, and ^ab^*P* < 0.05 means that the difference is statistically significant in the comparison between the groups.

## Data Availability

All data generated or analyzed during this study are included in this published article.
